# Water droplet behavior in between hydrophilic and hydrophobic surfaces and dust mitigation†

**DOI:** 10.1039/d2ra04845k

**Published:** 2022-10-10

**Authors:** Bekir Sami Yilbas, Abba Abdulhamid Abubakar, Johnny Ebaika Adukwu, Ghassan Hassan, Hussain Al-Qahtani, Abdullah Al-Sharafi, Muhammet Unal, Ammar Alzaydi

**Affiliations:** Mechanical Engineering Department, King Fahd University of Petroleum and Minerals (KFUPM) Dhahran 31261 Saudi Arabia bsyilbas@kfupm.edu.sa +966 3 860 4481; IRC for Renewable Energy and Power, King Fahd University of Petroleum and Minerals (KFUPM) Dhahran 31261 Saudi Arabia; K. A. CARE Energy Research & Innovation Center Dhahran 31261 Saudi Arabia; Turkish Japanese University of Science and Technology Istanbul Turkey; Engineering Faculty, Gazi University Ankara Turkey

## Abstract

An innovative method is introduced for environmental dust mitigation from a hydrophobic surface by a sessile water droplet. The sessile water droplet is located between two parallel plates having hydrophilic (at the top) and hydrophobic (at the bottom) states. The water droplet is located at the top hydrophilic plate, and the effect of the plate spacing on dust mitigation rate is examined. The droplet behavior is analyzed for different plate spacings and various droplet sizes using a high-speed camera. The fluid and the particle motions are simulated inside the droplet while adopting the experimental conditions. The findings demonstrate that the sessile droplet can effectively mitigate dust. Reducing the plate spacing increases the droplet meniscus diameter and enhances the dust removal rate. The surface tension force on the hydrophilic surface remains greater than that of the pinning force on the dusty hydrophobic surface even though the Magdeburg and surface tension forces contribute to the droplet pinning force on the hydrophobic dusty surface. Flow current is developed in the droplet fluid during the squeezing period, which considerably enhances the dust removal rate from the hydrophobic surface. The cleaned area increases with the droplet volume and plate spacing. Stria patterns are observed on the circumference of the dust-removed area. The present study provides a detailed analysis of a new method of dust removal from surfaces for self-cleaning applications.

## Abstract 2

An innovative method is introduced for environmental dust mitigation from a hydrophobic surface by a sessile water droplet.

## Introduction

One of the environmental impacts of climate change is the increased regularity of dust storms and dust settlement over surfaces across the Globe. Environmental dust is composed of many compounds such as silica, calcite, iron sulfate, sodium, potassium chloride, *etc.*^1^ These compounds can dissolve in water^2^ on rainy or humid days, and the resulting solutions can increase the dust particle pinning on surfaces.^3^ Among the major concerns of dust settlement on surfaces is the reduction in the performance of solar energy devices.^4^ Although several methods are proposed for dust mitigation from surfaces^5–8^, further studies are needed to develop efficient, self-sustained, and cost-effective dust mitigation methods. Self-cleaning surfaces for dust mitigation can offer some advantages over conventional cleaning methods, such as air blowing,^9^ water jet splashing,^10^ mechanical brushing,^11^ and others. This is because, in general, conventional methods either require compressed air, pressurized water, or mechanical displacement, which involve external electrical power preventing cost-effective operation. Self-cleaning generally requires a hydrophobic state on the surface where the settled dust particles are removed either by a sliding/rolling liquid droplet^12^ or by gravity.^13^ Since the hydrophobized surfaces have a low surface free energy and unique texture topology, the force of adhesion between the particles and the surface becomes low due to the weak van der Waals forces at the particle–surface interfaces. In addition, hydrophobic surfaces give rise to a Cassi–Baxter state on the surface where the surface repels the most common liquids, such as water. This gives rise to dust cleaning by the sliding and rolling motion of liquid droplets on the hydrophobized surface.^12^ The amount of mitigated dust depends on the droplet volume, the rate of droplet fluid infusion over dust surfaces, and droplet rolling velocity.^12,14^ Despite the rolling droplet mitigating dust from the surface, few dust residues can be observed on the surfaces,^14^ which raises several concerns for the quality of the cleaning process, particularly for cleaning of optical surfaces; nevertheless, further studies are required to improve the process. In addition, droplet rolling needs force to be created on a droplet, which overcomes the resisting forces *via* increasing the gravitational potential. Larger droplet volume results in an increased wetting area on the surface; consequently, the mitigated dust area becomes large. However, rolling droplets undergo wobbling because of gravitational potential, especially for the larger droplets.^15^ Hence, the striations occur along with the droplet path on the dusty surfaces,^16^ which adversely affects the uniformity of dust mitigated area, while suppressing the quality of the cleaning process. Nevertheless, developing a new and innovative dust mitigation mechanism becomes essential for efficient dust removal from hydrophobic surfaces.

In applications of surface self-cleaning, the main concerns are the surface topological characteristics and properties of the particles to be mitigated from the surfaces. The hydrophobic wetting state and the large size of the particles, which is larger than the micro/nanopillar spacings, become favorable for reducing particle adhesion and enhancing mitigation rates. Several methods are introduced toward hydrophobized surfaces for self-cleaning applications.^12,15,16^ The nano-composite coatings have become favorable in terms of cost-effective coatings. For example, surface coating with a nanolayer mixture of SiO_2_/N-TiO_2_ and hexadecyltrimethoxysilane (HDTMS) *via* spraying can produce a hydrophobic wetting state, which can be used in outdoor environments.^17^ However, the coating durability is limited to a few months of exposure in outdoor environments. The hydrophobic properties of coatings, such as self-healing, become an interest to increase the outdoor stability of the coating performance. In this case, the nanocomposites remain favorable for such coating applications.^18^ In addition, mesoporous titania–carbon (YbNTiO_2_@C) coating provides self-healing behavior on the surfaces; however, the high surface free energy of the coating material limits the practical application of dust mitigation from surfaces because of high pinning forces. One of the challenges of hydrophobic coating is the optical transparency as the coating is used in solar energy harvesting applications. The coating of glass surfaces by a transparent styrene–ethylene–butylene–styrene triblock copolymer (SEBS) can improve the optical transparency provided that the transmittance improvement is low, *i.e.*, within 75%.^19^ Introducing synthesized silica particles (F-SiO_2_) together with the functionalized carbon nanotubes (F-CNT) in the thin coatings can result in a hydrophobic state with self-healing ability.^20^ The resulting coating has a disadvantage for degradation under UV radiation; hence, it limits the possible usage in solar energy applications. Using a mixture of silicon carbide and chemicals such as dopamine and octadecylamine can improve the surface hydrophobicity and create self-cleaning ability on the coating surfaces. In this case, a stable nonfluorinated superhydrophobic mullite fabric, which is modified by silicon carbide nanowires, can be made on the surface^21^, providing that the coating surface becomes opaque to the optical spectrum. Hence, it cannot be used for self-cleaning the PV panel surfaces. Nevertheless, good biocompatibility, antibacterial, self-cleaning property, self-healing capacity, and stable functioning in outdoor environments remain the preference of this coating. Moreover, patterning the hydrophobic surfaces at nanoscale can provide the self-cleaning capability; however, further studies are needed to improve the optical transmittance.^22^

Among the alternative approaches for dust mitigation from surfaces is to utilize air humidity *via* self-cleaning by water vapor condensate on the hydrophobic surfaces. The condensate water on the hydrophobic surfaces forms droplets, which can be used for dust mitigation. However, additional arrangements are needed to increase the rate of condensation to form multiple droplets. One of the possible arrangements for increasing condensation is using fin and tube;^23^ however, this requires an additional arrangement for integrating such parts. Nevertheless, water condensation over the dusty hydrophobic surface remains critical for droplet formation. In the initial condensation phase, a liquid bridge is formed between the particles over the surface. The liquid infusion wets the particle surfaces in contact and, gradually, cloaks the particles. As the condensation progresses, a droplet can be formed over particles. With increasing droplet mobility, the particles in droplet fluids can be mitigated from the surface.^24^ However, the outdoor air condition is one of the major concerns, and rapidly changing conditions limit the method of such a self-cleaning process. Nevertheless, self-cleaning by rolling droplets over hydrophobic surfaces is among the promising dust cleaning methods. The droplet fluid infusion over dust surfaces and the cloaking of dust particles by the droplet fluid remains critical for the removal process by rolling droplets.^14,25^ On the other hand, during the process of cloaking, some salt compounds can dissolve in the droplet fluid while altering the droplet fluid properties.^25^ Hence, a fluid droplet composition changes to include the mixture solution composed of dissolved dust compounds and the droplet fluid. This modifies the droplet wetting length on the hydrophobic surfaces. In addition, as the mixture solution dries over the surface, it forms a layer between the dust particles and the hydrophobic surface. The dried layer enhances dust adhesion over the hydrophobic surface while preventing dust mitigation by rolling droplets.^26^ Hence, care is taken to increase the droplet mobility to avoid drying the mixture solution over the hydrophobic surfaces.

The droplet size needs to be kept large to increase the cleaned area over the surface. The large droplets suffer from wobbling because of gravitational influence giving rise to an unparalleled droplet path over the dusty surfaces while suppressing effective dust mitigation. Hence, a novel self-cleaning method must be introduced to minimize the ineffective self-cleaning of dusty hydrophobic surfaces. One of the novel approaches is to use a moving liquid droplet in between the hydrophilic and the hydrophobic surfaces. In this case, a hydrophilic surface can be located on the top, while a hydrophobic surface is at the bottom in the arrangement of parallel plates. Moreover, the hanging liquid droplet is attached to the hydrophilic surface in the gravitational direction. Yet, it remains attached to the hydrophilic surface because of the pinning force created by the surface tension, which remains larger than the droplet weight force.^27^ Reducing the spacing between the parallel situated hydrophilic and the hydrophobic plates enables the droplet to contact the hydrophobic surface at the bottom. Dust located over the hydrophobic surface is infused and cloaked by the droplet fluid across the wetted droplet area on the dusty hydrophobic surface.

The present study introduces a new (innovative) method of dust removal from surfaces for self-cleaning applications. The method can achieve self-cleaning with sessile (hanging) water droplets attached to movable hydrophilic plates; hence, dusty surfaces can be effectively cleaned at considerably lower workforce, energy, and water consumption costs. Hence, dust mitigation over the hydrophobic surface by a sessile droplet hanging down from the hydrophilic surface is examined. A fixture is assigned to accommodate two parallel plates consisting of hydrophilic and hydrophobic wetting states. The droplet is located at the top hydrophilic surface, which hangs down in the gravitational direction. Descending the top plate enables the droplet to touch the dusty hydrophobic surface. Consequently, this arrangement allows the droplet fluid to infuse and cloak the dust particles that settle on the hydrophobic surface. Once the top plate is moved up, the dust particles picked up by the droplet fluid are also moved up. Hence, the droplet behavior and dust mitigation rate from the hydrophobic surface are analyzed *via* a high-speed camera and an image tracking program. The study also includes the influence of plate spacing and droplet volume on the dust removal rates. In addition, a numerical study is incorporated to evaluate the droplet fluid behavior during squeezing and relaxing regimes of droplet motion within the parallel hydrophilic and hydrophobic surfaces. The velocity predictions provide information on the dust particle motion within the droplet.

## Experimental

Dust was collected from the outdoor glass surfaces in Dammam, *i.e.*, Eastern Province of Saudi Arabia. The collected dust was contained in sealed glass bottles. The dust was analyzed by electron microscope (JEOL 6460) and X-ray diffractometer (Bruker D8). Dust was mixed with distilled water to examine the solubility of some dust constituents in water. The resulting liquid solution was tested using a quadrupole inductively coupled plasma mass spectrometer (Thermo Scientific, XSeries 2). A computer-controlled fixture was designed to accommodate the glass plates in parallel while enabling the top plate to move vertically downward to the fixed stationary bottom hydrophobic plate. Fig. 1 shows the fixture and experimental setup. The bottom glass surface was hydrophobized by a dip-coating with functionalized silica nanoparticles. The silica nanoparticles were functionalized by preparing a mixture consisting of ethanol (14.2 mL), distilled water (1.2 mL), and ammonium hydroxide (24 mL) mixture.^28^ Afterwards, the tetraethyl orthosilicate (TOES) (1 mL TOES in 4 mL ethanol) was added. The surface wetting state was assessed using a Goniometer (Kyowa-DM 501). To observe and examines the droplet behavior in between the hydrophilic and hydrophobic surfaces, a high-speed camera (SpeedSense 9040) was accommodated, and it was operated at 5000 frames-per-second (fps), having an image resolution of 1280 × 800 pixels which corresponds to the dimensions, 14 μm × 14 μm. The uncertainty analysis was conducted for the data recorded. The uncertainty was estimated from:^29^1where *μ*_e_ is the average droplet wetting length (*x*) extracted from recorded data, *n* is the number of data, and *p*(*x*) is a probability distribution function whose diameter is obtained from the fitted Gaussian function to the data. The standard uncertainty was estimated to be within 3%. The bias uncertainty of 0.02 pixels was adopted because of the difficulties faced when assessing the small peaks in the function.

**Fig. 1:** The experimental setup images.

## Numerical modeling of dust particle motion within the compressed water droplet

Simulation of a compressed (squeezed) water droplet in between parallel plates is carried out. The flow equations and appropriate boundary conditions are considered in the simulations. The details of the mathematical formulations are given in the Appendix A. The flow field, temperature distribution, and particle trajectory are computed with the commercial finite element code, COMSOL Multiphysics. Three stages corresponding to droplet states before, during, and after droplet compression are considered in the simulations. The droplet geometries during these stages were recorded using the high-speed camera. Hence, the droplet geometries in the numerical model were reconstructed using the experimental data. The analysis adopts the 3D computation of the flow field and the temperature distribution with the dust particle trajectory. The boundary conditions adopted for the numerical simulation are shown in Appendix A (*i.e.*, Fig. 14a). The meshes are refined near the critical regions. The adopted mesh results in a grid-independent solution, as shown in the Appendix A (*i.e.*, Fig. 14b). Hence, the tetrahedral mesh with 129 342 elements is used in simulations based on the grid-independent test results. The time derivatives are discretized with the implicit scheme that utilizes time steps smaller than 10^−9^ s. Table 1 gives the properties used in the simulations.

**Table 1:** Material properties used in the simulations

Parameter	Water	Dust
Density (kg m^−3^)	838.5 + 1.4*T* − 0.003*T*^2^ + 3.7 × 10^−7^*T*^3^	2500 kg m^−3^
Viscosity (Pa s)	1.38 − 0.021*T* + 1.36 × 10^−4^*T*^2^ − 4.65 × 10^−7^*T*^3^	—
Surface tension (N m^−1^)	0.07275	—
Specific heat capacity (J kg^−1^ K^−1^)	12 010.15 − 80.41*T*^1^ + 0.31*T*^2^ − 5.38 × 10^−4^*T*^3^	82.68
Thermal conductivity (W mK^−1^)	−0.87 + 0.0089*T*^1^ − 1.58 × 10^−5^*T*^2^ + 7.98 × 10^−9^*T*^3^	2.05

### Initial conditions

Initially, the droplet and hydrophobic plates and droplet fluid are considered to be at 300 K and 295 K, respectively, as adopted in the experiments. The fluid velocity is initially zero, mimicking that of the sessile droplet. The initial pressure is taken as atmospheric (*i.e.*, 101.32 kPa), and the surrounding temperature is taken as 298 K.

### Boundary conditions

The wetted area between the hydrophilic plate and droplet (*i.e.*, top surface) is under a no-slip boundary, while a slip boundary condition is applied at the bottom surface, *i.e.*, the interface between the droplet and hydrophobic plate (Appendix A, Fig. 14a). A constant wall temperature is imposed along with the plates, and the plates were kept at 300 K. Natural convection is considered at the droplet–air interface. The Marangoni effect caused by the variation in surface tension with the temperature is also incorporated at the droplet–air interface.

## Results and discussion

Dust cleaning from a hydrophobic plate surface by a hanging water droplet is examined. An innovative design of two plates with different wetting states (*i.e.*, hydrophilic and hydrophobic) is introduced in the experiments to ensure the effective removal of dust particles. The sessile water droplet is formed on the hydrophilic surface facing towards the gravitational direction, and it is lowered to contact and wet the hydrophobic dusty surface. Later, it is raised to enable the removal of dust from the dusty plate surface. The droplet fluid motion during descending and ascending of the droplet is predicted and the dust particles behavior inside the droplet is examined. The mitigation rates and dust removed area are analyzed for different parallel plate spacings and droplet volumes.

### Hydrophobized surface and dust properties

Fig. 2a–c show the SEM (Fig. 2a) and AFM (Fig. 2b) images and the line scan (Fig. 2c), as obtained from AFM, of the hydrophobized surface, respectively. The coated surface demonstrates closely packed nanosized functionalized silica particles, which form clusters (Fig. 2a) on the surface. The clustered surface structures appear as nanopillars, which can be clearly seen from the surface line scan, as shown in Fig. 2c. The peaks in the line scan (Fig. 2c) demonstrate the nanosized pillars. The maximum pillar height is 325 nm, resulting in average surface roughness of about 155 nm. The surface roughness parameter (*r*), which measures the ratio of the area covered by pillars over the projected area, is estimated at 0.53. The equilibrium contact angle on the hydrophobic surface is calculated from high-precision Goniometer measurements.^30^ The droplet image on the goniometer screen is digitized, and the droplet circumference is fitted to a mathematical function. The crossing points of the horizontal line, resembling the droplet contact line, are located in the mathematical function. Since a slight tilt is observed between the fitted line and the actual contact line, the correction angle (*α*_BL_) is adopted when calculating the contact angle using the equation:^30^2where Δ*y* is the difference between the horizontal line and the center of the droplet resembled in the mathematical function, and *R* is the radius of the droplet as obtained from the mathematical function. The measurement of the contact angles is repeated fourteen times, and the estimated error is almost 3°.

**Fig. 2:** (a) SEM image of hydrophobic surface, (b) AFM image of the surface and line where line scan is conducted, and (c) surface line scan.

Fig. 3a shows the SEM images of the dust particles. In general, they are of different sizes and shapes. The average dust particle size is almost 1.2 μm. Some particles develop clusters and stick to the surface of the large ones (Fig. 3a). This may occur because of a long period of dust exposure to the Sun radiation, which can alter the dust charge forces.^3^ The shape can be categorized according to a geometric factor and the aspect ratio.^31^ The dust geometric factor is defined through  where *P* is the perimeter and *A* is the cross-sectional area. The aspect ratio is  where *L*_proj_ is the longest length on the dust particle projection.^2^ It is worth mentioning that for the dust particles resembling a circular shape, the aspect ratio and the shape factor approach one, and the dust particle becomes almost circular. This occurs mainly for the particles having sizes below the average dust particle size. The median of the aspect ratio is about 2.8 for particle sizes greater than 4 μm, while it reduces to 1.3 for the average size of particles (∼1.2 μm). Furthermore, a dust particle is composed of different elements and compounds. Fig. 3b shows the XRD spectrum, while Table 2 gives the EDS data of dust. The compounds in the XRD graph indicate that peaks are due to silica (SiO_2_), gypsum (CaSO_4_), salt (NaCl), hematite (Fe_2_O_3_), and calcite (CaCO_3_). However, the elemental composition changes slightly as the dust particle size increases (>1.2 μm); hence, chlorine, sodium, and potassium reduce for large dust sizes (Table 2). Dust cannot mitigate from the hydrophobic surface unless the droplet fluid infuses over its surface with a spreading coefficient higher than zero. The spreading coefficient (*S*) can be: *S* = *γ*_s_ − *γ* − *γ*_s–L_, here, *γ*_s_ is the dust particle surface free energy, *γ* is the droplet fluid surface tension, and *γ*_s–L_ is the interfacial tension.^31^ Since the droplet fluid is water, the spreading coefficient can easily be calculated. Dust surface free energy and interfacial resistance become: *γ*_s_ = 114.5 ± 5.5 mJ m^−2^ and *γ*_s–L_ = 20.55 mJ m^−2^.^25^ The surface tension of the distilled water is 0.072 N m^−1^, and the spreading coefficient becomes *S* = 21.95 mJ m^−2^. This demonstrates that the water infuses the dust surfaces and wets the particles. Fig. 4 shows the cloaking (infusion) velocity of the droplet fluid over a dust particle with time. The infusion rate over the dust surface is determined by measuring the droplet fluid cloaking velocity. The cloaking velocity reduces with increasing time, which is consistent with the early.^25^ It is worth mentioning that the cloaking velocity depends on the shape of a particle;^25^ however, this dependence becomes weak because of the small dust particle sizes. In general, the temporal decay of cloaking velocity follows an exponential form as ∼_*K·*e*^−mt^*_, where *K* is the initial velocity, which is considered to be constant, *m* is related to the power of the decay rate.^32^ The tests carried out for evaluating the cloaking velocity are repeated over ten times, incorporating the different dust particle sizes and shapes; the error estimate is about 12%, with *m* being within the range of *m* = ¼1/*s* for all measurements. Moreover, the shear, surface tension, and gravitational forces influence the rate of the droplet fluid cloaking over the dust surface. Since the shear and gravitational forces have an adverse effect while surface tension force promotes the water cloaking process, the ratio of shear to surface tension forces (Ohnesorge number:  where *μ* is viscosity, *ρ* is the density, and a represents the particle size), and the ratio of weight over the surface tension force (Bond number:  where Δ*ρ* is the density difference, *g* is the gravitational acceleration) remain important. The dust particle size used for the cloaking velocity assessments varies from 1 μm to 10 μm. This leads to the Ohnesorge number variation in between 1.05 × 10^−4^ to 0.33 × 10^−4^ while the Bond number varies in between 1.36 × 10^−7^ to 1.23 × 10^−5^. This demonstrates that the shear force remains dominant during the cloaking period compared to the weight force. Moreover, the time corresponding to the complete infusion of the droplet fluid over the dust particle is about 0.245 ms for the average dust particle size (1.2 μm) as predicted in previous studies.^31^ Moreover, the salt compounds present in the dust particles can dissolve in water during the infusion, affecting the droplet fluid's properties such as pH, surface tension, and density. A solution is extracted from the dust and water mixture and analyzed using inductively coupled plasma spectrometry (ICP) and acidity measurements. The pH of the droplet fluid increases from 6.2 to 8.6, demonstrating the fluid's acidity is reduced because the alkaline (NaCl and KCl) and alkaline earth metal salts (CaCl) dissolves in the water droplet. However, the droplet surface tension, due to the dissolution of alkaline salts, changes slightly, as shown in Table 3. The extracted ICP data is also shown in Table 4.

**Fig. 3:** (a and b) SEM image of dust demonstrating various shapes and clustering of the dust particles and (c) X-ray diffractogram.

**Table 2:** Dust sizes and elemental compositions (wt%)

	Si	Ca	Na	S	Mg	K	Fe	Cl	O
Size ≥1.2 μm	11.7	8.2	2.1	1.3	2.4	0.8	1.2	0.4	Bal.
Size <1.2 μm	10.3	7.4	2.7	2.2	1.4	1.2	1.1	1.1	Bal.
Dust residues	9.5	7.1	1.9	1.4	1.9	1.1	0.9	0.9	Bal.

**Fig. 4:** Water cloaking velocity of dust particle with time.

**Table 3:** Variation of droplet surface tension with dust concentration

Concentration (weight%)	Surface tension (N m^−1^)
0	0.0720
5	0.0724
10	0.0735
15	0.0741
20	0.0741

**Table 4:** ICP data for the dust–water mixture. Unit is ppb

Ca	Na	Mg	K	Fe	Cl
308 900	45 400	69 500	34 500	1800	36 600

### Dust mitigation

As the plate spacing reduces, the droplet contact angle and the wetting length change. Since the surface tension force is related to the pinning of the droplet, droplet expansion on the hydrophobic surface becomes suppressed during the top plate squeezing. The vertical component of the surface tension force is ∼−π*D*_w_*γr*sin *θ*, here, *D*_w_ is the wetted droplet diameter, *r* is the roughness parameter, and *θ* is the average droplet contact angle. The droplet contact angle changes with the plate spacing, as demonstrated in Fig. 5a and b . As the plate spacing reduces, the average contact angle decreases and the resistance created for the droplet expansion also reduces over the surface. The Laplace pressure increases in the droplet fluid as the plate spacing reduces, which results in the radial expansion of droplets, *i.e.*, the droplet width increase. In addition, the contribution of the surface tension to the droplet wetting diameter extension also changes. This limits the value of the maximum droplet wetting diameter. Fig. 6a and 7b show the wetting length of the droplet (=π*D*_w_, *D*_w_ is the wetting diameter) at the bottom surface (hydrophobic) with the droplet volume for two plate spacings. The wetting length increases with the droplet volume for the plate spacing of 1 mm. The wetting length attains slightly smaller values on the dusty hydrophobic surface than on the clean surface. This is attributed to the change in the droplet surface tension force on the dusty surface (Table 3). In addition, the percentage of wetting length decay, due to the change of plate spacing from 1 mm to 2 mm, is 54% for 30 μL droplets; however, the decline becomes about 38% for 60 μL droplets. Hence, the reduced plate spacing has a more significant effect on the wetting length. On the other hand, as the plate spacing reduces further, the droplet pins over the hydrophobic plate and attaches to the hydrophobic surface as the plate spacing is increased through the upper motion of the top hydrophilic plate. This situation can be observed from Fig. 7, where the droplet attaches over the hydrophobic surface at different plate spacings. Attachment of the droplet is related to the nanosized cavities on hydrophobic surface texture. Hence, squeezing the droplet in between the plates, air occupying the cavities is purged out by the droplet bottom surface while creating the vacuum sites in this region. The droplet develops a curvy arc meniscus at the top of the texture. As the squeezing ends and the top plate is progressing towards increasing the plate spacing, the vacuum created in the nanocavities holds the droplet bottom surface through the Magdeburg effect. The force created due to the Magdeburg effect can be written as:^33^3here *n*_*p*_ is the number of gaps created by four consecutive pillars where the air gap is created in between them, ma is the mass of air occupying the gap, *R* is the universal gas constant, and *T* is the air temperature of air occupying the gap, *b* is the maximum pillar height, *b*_0_ is the height of the pillar up to the point of droplet fluid inflection in between two consecutive pillars. The fluid inflected from the droplet bottom into the texture pillars gap cannot occupy the pillars gap totally, and the height of inflected fluid (*b* − *b*_0_) can be derived from the force balance relation.^33^ Using the equation introduced in the previous work^33^ and using the AFM line scan data, the liquid inflection depth can be estimated. Hence, the average spacing between two consecutive pillars is about ∼2 μm (Fig. 2c), and the average pillar height is ∼100 nm (Fig. 2c), the fluid inflection height in the gap between the consecutive pillars can be estimated as 30 nm during squeezing the droplet, which is almost 1/3 of the height of the pillar. Since the wetted diameter for 50 μL droplet is about 2.23 mm and the wetted area is about 3.9 mm^2^. The average area covered by the four pillars forming a cavity is about ∼4 × 10^−6^ mm^2^, and the number of gap sites  where *k* is the percentage of the cavity that traps the air within ∼4 × 10^−6^ mm^2^ cavity (*k* is taken as 1%), *n*_f_ is the fraction of area covered by the solid pillar area (1 − *n*_f_) is about 0.2 as estimated from the surface line scan (Fig. 2c), by *A*_wetted_ is the wetted area of the droplet corresponding to the minimum plate spacing, *A*_pillars_ is the four consecutive pillars forming the air gap yields about *n*_p_ = 2.83 × 10^2^. Hence, setting the air temperature as 25 °C, air gas constant *R* = 287 J kg^−1^ K^−1^, *b* is ∼100 nm, *b*_0_ is ∼70 nm, and *n*_p_ ∼ 2.83 × 10^2^, and Ma ∼ 9.6 × 10^−20^ kg, the Magdeburg force created below the droplet yields about −5.57 × 10^−4^ N. However, the vertical component of the surface tension force for the droplet attaching at the hydrophilic surface (top) surface is ∼π*D*_wT_*γ*sin *θ*_T_, here *D*_wT_ (∼4.8 mm) is the wetted droplet diameter for the top surface, *θ*_T_ (∼75°) is the average droplet contact angle for the top surface, when the plate spacing is at the minimum. Hence, inserting the values, the vertical component of the surface tension force on the top surface yields 1.07 × 10^−3^ N. In addition, the vertical component of the surface tension force for the bottom (hydrophobic) surface is about −1.35 × 10^−4^ N. Therefore, the vertical force balance yields a positive net force, *i.e.*, the summation of the magnitude of the vertical component of Magdeburg and the surface tension force on the bottom plate (hydrophobic) is less than the vertical component of the surface tension force created at the top surface (hydrophilic). In addition, the magnitude of the Magdeburg force is greater than that of the vertical component of the surface tension force. This causes droplet stretching on the hydrophobic surface while moving the top surface from the squeezed state of the plates, *i.e.*, despite enlarging the plate spacing, the bottom surface pinning continues, and stretching of the droplet occurs as the plate spacing is further enlarged (Fig. 7). Consequently, care is taken to avoid droplet attachment on the hydrophobic surface through proper setting of the plate spacing during the squeezing action. Fig. 8 shows optical images of droplets in between the hydrophilic (top) and hydrophobic (bottom) plates for different distances between the parallel plates (plate spacing). The droplet picks up dust particles as the plate spacing is enlarged. The droplet-wetted length on the dust surface increases as the plate spacing reduces, allowing the droplet fluid to wet more dust particles on the bottom surface. Hence, the dust picked up increases as the plate spacing reduces. However, the amount of dust picked up is not linearly varying with the plate spacing (Fig. 9), in which the area of dust removed from the bottom surface with plate spacing is given for various droplet sizes. In addition, Fig. 10 depicts the optical images of the dust-removed areas from the bottom surface. The area of dust removed reduces as the plate spacing increases and the change of area increase becomes more apparent for small plate spacings (<1.5 mm) for all droplet volumes considered. The dust removal rate from the bottom surface increases with increasing droplet volume due to increasing wetting length of the droplet (Fig. 6). Striation occurs around the circumference of the dust removed area due to the infusion of a droplet over the dust particles surfaces. Moreover, only the dust particles that are completely cloaked by the droplet fluid are picked up.^31^ Since the dust particle size varies, this enables some of the small dust size particles wetted by the droplet fluid and some large particles to remain partially wetted around the meniscus of the droplet. The partially and/or unwetted particles in the circumference of the droplet meniscus are left over the dusty surface while appearing as part of the dust striations. In addition, very few dust particles remain over the area cleaned, which can be observed from Fig. 10. Although they are few, the dust residues are mainly observed for small plate spacings. This indicates that the residues can be related to the adhesion of the water droplet at the interface of the dusty surface because of droplet fluid inflection in nanocavity sites at low plate spacings. Nevertheless, dust residues are few and do not significantly affect the display of the total area cleaned.

**Fig. 5:** Contact area of droplet on dusty surface with plate spacing and optical image of two squeezed water droplet and contact angle variation with plate spacing.

**Fig. 6:** Droplet wetting length (π*D*_w_) on the clean and dusty hydrophobic surface for two plate spacings: (a) plate spacing is 1 mm, and (b) plate spacing is 2 mm.

**Fig. 7:** Side view of 40 μL droplet: (a) droplet away from dusty hydrophobic surface, (b) droplet touching dusty hydrophobic surface and plate spacing is 1 mm, (c) droplet partially moved up and droplet fluid picks up some dust, and (d) and (e) droplet moved from the dusty hydrophobic surface and small droplet section temporarily attaches hydrophobic surface.

**Fig. 8:** Side view of droplet in between the top hydrophilic and bottom dusty hydrophobic plates for different droplet volumes: (a) 40 μL, (b) 50 μL, and (c) 60 μL. The arrow shows the motion of the top hydrophilic plate.

**Fig. 9:** Area of dust removed with plate spacings for different droplet volumes and two different plate spacings: (a) 1 mm plate spacing, and (b) 2 mm plate spacing.

**Fig. 10:** Optical images of top view of dust removed areas for different plate spacings and various droplet volumes. Dark region shows the dust removed area.

Fig. 11 shows 3D predictions of flow velocity (Fig. 11a), pressure (Fig. 11b), and temperature (Fig. 11c) of 40 μL droplet for 1 mm minimum plate spacing after squeezing in between the hydrophilic (at the top) and hydrophobic (at the bottom) plates. The droplet fluid under compression creates the flow circulation structures within the droplet interior (Fig. 11a). The velocity attains almost the maximum at the droplet fluid, interfacing the hydrophobic surface in the region away from the centerline. In the proximity of the centerline at the interface, a stagnation zone is created, and the droplet radial extension increases the flow velocity near the stagnation zone. The pressure attains larger values in the droplet fluid close to the hydrophobic surface than that of the hydrophilic top surface (Fig. 11b), as observed from Fig. 11c. This is attributed to the hydrostatic effect of the droplet fluid due to the droplet height, and resistance to the radial extension on the hydrophobic surface because of the surface tension force. During the droplet squeezing, the temperature of the fluid increases slightly (Fig. 11c) and the temperature difference between the upper (close to top plate) and lower (close to bottom plate) sections of the droplet fluid can contribute to the flow field because of surface tension gradient, *i.e.* the Marangoni currently can be created; however, since the temperature difference is small, the flow current intensity is expected to be small. Fig. 12a and b show velocity and pressure variation along the horizontal line located in the droplet fluid for different periods of 40 μL droplet squeezing. The velocity magnitude remains higher near the droplet-free surface region. However, velocity reduces considerably at locations where the center of circulation occurs. Since the rotating flow structures have a counter-rotational motion, velocity reaches the maximum at the interfacial boundaries of the rotating structures. The peak value of velocity demonstrates temporal behavior along with the horizontal line (Fig. 11a). Temporal behavior is attributed to the transient fluid motion created during the droplet squeezing periods. Nevertheless, the magnitude of the peak velocity remains within the order of mm s^−1^. The pressure variation along the horizontal line changes with small magnitudes. However, the pressure change is notably high with time in the droplet fluid. Hence, droplet squeezing creates a fluid motion changing with time. The droplet fluid pressure and velocity change rapidly in the early squeezing period, *i.e.*, the radial droplet expansion influences the surface tension force. The pressure distribution within the fluid and local high-pressure region is formed within the proximity of the droplet–surface interface (Fig. 11b). Fig. 13 shows the dust particle trajectory at different periods. It can be seen that the particles are moved into the droplet interior under the shear force. However, the particles remain in the interfacial region of the droplet fluid until they are cloaked. The flow currents, developed because of dynamic change of the fluid pressure during squeezing and the Marangoni, carry the dust particles towards the droplet interior. However, the Marangoni force over the local convection force created by the rapid change of the fluid pressure is related to the velocity ratio, *i.e.*, the force ratio is  here *v*_M_ is the flow velocity due to Marangoni current, and *v*_p_ is the flow velocity due to pressure change. In addition, the force ratio is the twice order of the pressure coefficient over the droplet Weber number *i.e.*,  where *a* is the droplet size (droplet diameter). Hence, using the pressure predictions,  becomes about 0.60. Since the force ratio is similar to the square of velocity ratios  this indicates that the Marangoni influence becomes less important than that of the pressure variation created during the squeezing of the droplet for dust mitigation/motion. The buoyancy force can ease dust mitigation inside the droplet fluid. This is particularly true for some particles, which have low densities.^34^ Moreover, the local Reynolds number ( where *v* is the droplet fluid flow velocity, *a* is the droplet size, and *μ* is the fluid viscosity) plays a significant role in the particles to be carried away by the flow pattern created inside the droplet. For low Reynolds number flow, the particle Stoke's number is vital to the particle motion inside the droplet fluid. From the simulations, the average flow velocity is bout 5 × 10^−4^ m s^−1^, fluid density is 1000 kg m^−3^, viscosity is 8.9 × 10^−4^ Pa s, the local Reynolds number in the droplet fluid yields about 1.13 for the droplet height of 2 mm in between the plates. The behavior of the particles at low Reynolds number flow can be governed by the particle Stokes number, which can be written as  here *ρ*_p_ is the particle density, *d*_p_ is the particle diameter, *l*_0_ is the characteristics dimension of the flow domain (can be considered as the droplet height, a). Inserting the particle density (∼2800 kg m^−3^),^34^ the average particle size (1.2 μm), the average fluid velocity predicted (5 × 10^−4^ m s^−1^), and fluid viscosity (8.9 × 10^−4^ Pa s), and characteristic size of the flow domain (2 × 10^−3^ m), the particle Stoke number becomes 0.126 × 10^−3^, which is much smaller than 1, *i.e.* Stk ≪ 1. Hence, the flow streams inside the droplet fluid influence the dust particle motion.^35^ Hence, the flowing current developed enhances the dust rate from the interfacial region of the droplet fluid.

**Fig. 11:** 3D distribution of velocity, pressure, and temperature in 40 μL droplet for plate spacing of 1 mm: (a) velocity inside droplet, (b) pressure inside droplet and (c) temperature inside droplet.

**Fig. 12:** Velocity and pressure variation along the horizontal line located at 0.5 mm from hydrophobic surface for different periods and plate spacing of 1 mm: (a) velocity distribution, and (b) pressure distribution.

**Fig. 13:** Velocity and distribution of dust particles inside 40 μL droplet fluid obtained from simulations at different periods for plate spacing of 1 mm.

**Fig. 14:** (a) Boundary conditions and solution domain, (b) grid used, and (c) mesh convergence test results predicted for flow velocity along a horizontal line located at 1 mm from hydrophobic bottom surface.

## Conclusion

An innovative method for removing a hanging water droplet is introduced, and the droplet wetting states in between parallelly located hydrophobic and hydrophilic plates are examined. The water droplet formed on the hydrophilic plate (located at the top) is descended towards the hydrophobic plate (located at the bottom). The droplet squeezing motion in between parallel plates alters the droplet shape and the wetting length. Since dust is spread over the surface, the droplet fluid infusion causes the mitigation of dust from the hydrophobic plate surfaces. As the top plate has raised, the droplet attached to the top plate detaches from the bottom surface while mitigating the dust particles. As the plate spacing reduces beyond 1 mm for droplet volumes larger than 40 μL, inflection of the droplet fluid creates a Magdeburg force because of the displacement of air captured inside the microcavities during the droplet squeezing. This enhances the droplet pinning over the surface while ascending the top plate. The vertical Magdeburg force component created on the hydrophobic surface (5.57 × 10^−4^ N) remains less than the vertical surface tension force component (1.07 × 10^−3^ N) on the hydrophilic top cover for the plate spacing of 1 mm. Hence, dust infused into the droplet fluid is mitigated from the hydrophobic bottom surface by the droplet during the top plate ascending. Moreover, the dust mitigated area on the hydrophobic surface increases with the droplet volume and plate spacing. The droplet wetting length and cleaned area do not vary linearly with the plate spacing, especially for the large volume droplets. The stria patterns are observed on the circumference of the dust removed area, which is attributed to incomplete infusion of the droplet fluid over large size dust particles located in the meniscus of the droplet on the hydrophobic surface. The dust particles, which are completely infused by the droplet fluid, can be mitigated from the hydrophobic surface. However, few dust residues remain in the dust mitigated surface region due to droplet fluid pinning under the Magdeburg forces created at the liquid–surface interface. The droplet fluid pressure and the flowing current created in the interface region of the droplet change rapidly in the early squeezing period. This enables carrying the dust particles from the droplet interface to the droplet interior. The present study provides a detailed analysis of a new method introduced for dust removal from hydrophobic surfaces and gives insight into the droplet pinning forces due to the Magdeburg effect created in nanocavities.

## Appendix A: flow field formulation incorporating the particles

The equations governing the flow field are continuity, momentum, and energy, which are treated individually. The continuity equation is:

4 ∇*v̄* = 0

here: *v̄* represents the velocity vector.

The momentum equation can be expressed as:5here: *ρ* is fluid density, *p* is gauge pressure, *p*_0_ is hydrostatic pressure, *μ* is viscosity, *g* is gravity, *T* is temperature,  denotes the contribution of the dust particle motion to the total volumetric force acting on the fluid, *n* is the total number of dust particles, *r̄* is the spatial coordinate, *δ* is the Dirac delta function, and *s̄*_j_ is the position vector of the particles.

Density variation due to the thermal expansion of water can be represented as:

6 *ρ* = *ρ*_0_(1 − *β*(*T* − *T*_0_))

here: *β* is coefficient of thermal expansion, *ρ*_0_ is reference density, and *T*_0_ is reference temperature.

The energy equation predicts the distribution of temperature within the droplet fluid. Adopting natural convection on the free droplet surface, the energy equation becomes:7here: *C*_p_ is specific heat capacity and *k* is thermal conductivity.

The Bond number (Bo) can be represented as:8here: *γ* is the surface tension, *m* is length scale taken as:  with *V*_l_ is the droplet volume and *r*_w_ is the wetting radius.

The Grasshoff number (Gr) is:9here: Δ*T* is temperature difference and *ν*_0_ is the kinematic viscosity.

The Marangoni number (Ma) is also represented as:10here: *α* represents the thermal diffusivity.

The Merve number representing the ratio of gravitational force over surface tension force, which is given as:^36^11

The movement of bubble and dust particles within the droplet is governed by the second law of Newton, *i.e.*:12where: *m*_d_ is the mass of dust particles, and *F*_t_ is the total force acting on the bubble/particle.

The total force acting on the particle yields:

13 *F̄*_t_ = *F̄*_b_ + *F̄*_g_ + *F̄*_d_

here: buoyancy force is  gravitational force is *F*_g_ = *m*_d_*gi*, and drag force is *ρ*_d_ is the density of the particle, *τ*_d_ is particle velocity response and *V*_d_ is the velocity of the particle. The particle velocity response is given by:14

## Conflicts of interest

There are no conflicts to declare.

## Supplementary Material

RA-012-D2RA04845K-s001
